The article "Expression and clinical significance of hypoxia-inducible factor 1α, Snail and E-cadherin in human ovarian cancer cell lines" was retracted in 2025. Reasons: plagiarized data; overlap with other authors' work; concerns about the data.

# Expression and clinical significance of hypoxia-inducible factor 1α, Snail and E-cadherin in human ovarian cancer cell lines

**DOI:** 10.3892/mmr.2015.3786

**Published:** 2015-05-14

**Authors:** YAN ZHANG, NINA FAN, JING YANG

**Affiliations:** 1 Department of Gynaecology and Obstetrics, Renmin Hospital of Wuhan University, Wuhan, Hubei 430060, P.R. China; 2 Department of Gynaecology and Obstetrics, Hubei Xinhau Hospital, Wuhan, Hubei 430060, P.R. China

**Keywords:** hypoxia-inducible factor 1α, zinc finger transcription factor, E-cadherin, epithelial-mesenchymal transition, ovarian cancer

## Abstract

The aim of the present study was to investigate the expression and clinical significance of hypoxia-inducible factor 1α (HIF-1α), Snail and E-cadherin in ovarian cancer. The expression levels were assessed in a number of ovarian cancer cell lines and ovarian cancer tissues, and correlations between the expression of the three proteins and clinical pathological factors were analyzed. Transwell assays showed that the invasive ability of the ovarian cancer cell lines SKOV3 and ES-2 were significantly higher than those of TYK and 3AO (P<0.01). Furthermore, the expression levels of HIF-1α and Snail in SKOV3 and ES-2 were significantly higher than those in TYK and 3AO, whereas the expression levels of E-cadherin in SKOV3 and ES-2 were significantly lower than those in TYK and 3AO (P<0.05). In ovarian cancer tissues, the expression levels of HIF-1α, Snail and E-cadherin were correlated with clinical pathological factors (P<0.01); furthermore, there was a positive correlation between the expression levels of HIF-1α and Snail (r=0.231; P=0.021), and a negative correlation between the expression levels of Snail and that of E-cadherin (r=−0.225; P=0.028). HIF-1α was suggested to be able to suppress the expression of E-cadherin by upregulating Snail, thus serving an important role in invasion and metastasis of ovarian cancer.

## Introduction

Ovarian cancer is a common malignant tumor of the female reproductive system and has one of the highest mortality rates out of all gynecological malignancies, presenting a serious threat to women's health and lives (1). Previous studies have observed that the transformation of epithelial cells to mesenchymal cells (epithelial-mesenchymal transition; EMT) is important in various stages of development of various types of cancer, including colon, skin, breast, ovarian and pancreatic cancer, hepatocellular and lung adenocarcinoma. In particular, EMT has been reported to promote invasion and metastasis (2). EMT occurs in specific physiological and pathological conditions, including the basic process of biological embryonic development, organ formation and cell migration, and the early stages of the tumor metastasis cascade reaction as a key factor in the process of invasion and metastasis (2).

The article "Expression and clinical significance of hypoxia-inducible factor 1α, Snail and E-cadherin in human ovarian cancer cell lines" was retracted in 2025. Reasons: plagiarized data; overlap with other authors' work; concerns about the data.

EMT involves multiple signaling pathways and a variety of complex molecular mechanisms. Previous studies have demonstrated that the Snail transcription factor functions as an inducer of the EMT during embryonic development, and Snail is able to directly inhibit the expression of E-cadherin to regulate EMT (3,4). E-cadherin is a calcium-dependent glycoprotein distributed in the epithelial tissue, which mediates homogeneous adhesion between cells. As a typical epithelial phenotypic marker, it is an important molecule in the maintenance of the epithelial phenotype; the reduction and loss of E-cadherin expression have been reported to result in a decline in cell adhesion (5,6). E-cadherin is an inhibitory factor for the malignant transformation of tumors, invasion and metastasis; the functional loss of adhesion in cell-cell contacts mediated by E-cadherin is a rate-limiting step of cell dedifferentiation and invasion (7,8). Previous studies have observed that in a number of malignancies, including ovarian cancer, certain factors are able to regulate the expression of E-cadherin by regulating Snail, thus affecting the occurrence of tumor cell invasion and metastasis (7,8).

Hypoxia is a common characteristic of the vast majority of malignant tumors, particularly solid tumors (9). However, the association between the hypoxic microenvironment and Snail genes in tumors remains to be elucidated. Hypoxia-inducible factor lα (HIF-1α) serves a key role in the regulation of the intracellular oxygen metabolism and its overexpression is closely associated with malignant behaviors, including tumor cell proliferation, invasion and metastasis (9). Luo *et al* (10) identified a hypoxia-response element (HRE) at the Snail gene promoter sequence using luciferase reporter gene and ChIP assays. Through a combination of HRE sites, HIF-lα directly regulates Snail transcription and expression, indicating that the Snail gene contains the structural basis of hypoxia regulation.

Therefore, the present study aimed to investigate the expression and clinical significance of HIF-1α, Snail and E-cadherin in the human mucinous ovarian cancer cell line 3AO, the serous ovarian cancer cell line SKOV3, the human clear cell ovarian cancer cell line ES-2 and the undifferentiated human ovarian cancer cell line TYK, as well as in ovarian cancer tissues.

## Materials and methods

### Cell lines

The serous ovarian cancer cell line SKOV3 was purchased from the Cell Center of the Institute of Basic Medical Sciences, Chinese Academy of Medical Sciences (Beijing, China), the mucinous ovarian carcinoma cell line 3AO was purchased from the Central Laboratory of Tianjin Medical University (Tianjin, China), the human clear cell ovarian cancer cell line ES-2 was purchased from Shanghai Aiyan Research Biotechnology Co., Ltd. (Shanghai, China) and the undifferentiated ovarian cancer cell line TYK was provided by the Cancer Center of Qilu Hospital at Shandong University (Jinan, China).

The article "Expression and clinical significance of hypoxia-inducible factor 1α, Snail and E-cadherin in human ovarian cancer cell lines" was retracted in 2025. Reasons: plagiarized data; overlap with other authors' work; concerns about the data.

### Patient samples

The ovarian cancer tissues were obtained via surgical resection from 182 patients with ovarian cancer at Renmin Hospital of Wuhan University between February 2010 and 2012 and the tissue was divided into histological grades I, II and III (11). The patients were 32–57 years of age and surgical resection was performed 1–6 months post-diagnosis. The inclusion criteria for the present study were as follows: Female, ≥18 years, confirmed histologically as Stage I–III epithelial ovary primary cancer, white blood cell content ≥3,000/*µ*l, absolute neutrophil count ≥1,500/*µ*l, hemoglobin content ≥9 g/ml and platelet count ≥100,000/mm^3^. Patients with other medical conditions, which precluded the study were excluded depending on the opinion of the authors. The present study was approved by the ethics committee of Renmin Hospital of Wuhan University (Wuhan, China) and written consent was obtained from all patients.

### Main reagents

RPMI-1640 culture media and trypsin were purchased from Gibco-BRL (Invitrogen Life Technologies, Carlsbad, CA, USA). Fetal calf serum was purchased from Hangzhou Evergreen Biological Engineering Materials Co., Ltd. (Hangzhou, China), MTT was purchased from Amresco LLC (Solon, OH, USA) and dimethyl sulfoxide was purchased from Sigma-Aldrich (St. Louis, MO, USA). The Transwell chamber was purchased from Corning-Costar (Corning, NY, USA), the artificial basement membrane (Matrige1) was purchased from BD Biosciences (Franklin Lakes, NJ, USA), the reverse transcription polymerase chain reaction (RT-PCR) kit (Access Quick RT-PCR system) was purchased from Promega Corporation (Madison, WI, USA); anti-human Snail and anti-human E-cadherin mouse monoclonal antibodies were purchased from Santa Cruz Biotechnology, Inc., (Dallas, TX, USA) and the prestained protein marker (cat. no. BRP-125) was purchased from SBS Genetech (Beijing, China).

### Cell culture

The cells were cultured in RPMI-1640 medium supplemented with 10% fetal bovine serum, 2 mmol/l glutamine, 100 U/ml penicillin and 100 U/m1 streptomycin, all purchased from Invitrogen Life Technologies. Cells were cultured in incubators at 37°C in humidified air containing 5% CO_2_.

### Cell invasion assay

The Transwell chamber assay was applied to detect cancer cell invasion (12). The number of cells transgressed through a polycarbonate membrane was counted under the light microscope (CKX41-A32RC; Olympus, Tokyo, Japan; magnification, x400), and the relative number of invasive cells represented the tumor cell invasion. The number of cells was counted within six random fields of view, the average was deduced and three samples were counted for each group.

The article "Expression and clinical significance of hypoxia-inducible factor 1α, Snail and E-cadherin in human ovarian cancer cell lines" was retracted in 2025. Reasons: plagiarized data; overlap with other authors' work; concerns about the data.

### Total RNA extraction and identification

Total RNA extraction was conducted using TRIzol reagent (Invitrogen Life Technologies) in accordance with the manufacturer's instructions for the kit used (Huamei Company). Subsequent to extraction of the RNA, the concentration and purity of the RNA sample was determined by measuring the optical density within 6 h.

### RT-PCR using the two-step method

Total RNA extraction was performed in accordance with the manufacturer's instructions for TRIzol. Synthesis of first-strand cDNA was performed in accordance with the kit. Briefly, l *µ*l oligo (dT) were added to 2 *µ*g total RNA and heated at 70°C for 5 min. A total of 5 *µ*l 5X avian myeloblastosis virus (AMV) buffer, 2.5 *µ*l desoxyribonucleotide triphosphate (10 mmol/l), 1 *µ*l AMV-RT (10 U/*µ*l), l *µ*l RNasin (40 U/*µ*l; Promega Corp.) and diethylpyrocarbonate-treated water were then added to a final volume of 25 *µ*l, mixed and reacted at 42°C for 60 min.

The PCR primers were synthesized by Sangon Biotech Co., Ltd. (Shanghai, China; Table I). PCR cycling conditions were as follows: 94°C for 2 min, 35 cycles of 94°C for l min and 58°C for 1 min, followed by extension at 72°C for l min, on a GeneAmp PCR system 9600 (Applied Biosystems). Expression levels were calculated relative to GAPDH levels, which acted as the endogenous control. The PCR products then underwent 1% agarose gel electrophoresis and were observed under an ultraviolet lamp and images were captured on a Bio-Rad VersaDoc 3000 Imaging system (Bio-Rad). Image J software (NIH, Bethesda, MD, USA) was used for grey value analysis.

### Western blot analysis

The total protein was extracted from the cells and quantified using a bicinchoninic acid assay (Pierce Biotechnology, Inc., Rockford, IL, USA). Equal quantities (40 *µ*g) of protein sample were loaded, separated by electrophoresis at 120 V for 1.5 h and transferred onto polyvinylidene difluoride (PVDF) membranes (Bio-Rad) at 90 mA for l2–16 h at 4°C. The film was then stained with 0.1% Ponceau S (Bio-Rad) to determine the location of the transfer efficiency and protein marker. The PVDF membranes were blocked by freshly prepared blocking buffer (1X Tris-buffered saline, 5% skimmed milk and 0.05% Tween-20; Sigma-Aldrich, St. Louis, MO, USA) prior to incubation with the primary antibodies, mouse anti-human HIF-1α (cat. no. sc-13515), anti-human Snail (cat. no. sc-393172), anti-human E-cadherin (cat. no. sc-21791), anti-human GAPDH (cat. no. sc-365062) monoclonal antibodies (Santa Cruz Biotechnology) and rabbit anti-mouse IgG horseradish peroxidase conjugated secondary antibody (sc-358914) (Santa Cruz Biotechnology), according to the manufacturer's instructions. This was followed by incubation with the secondary antibody and the protein was visualized using an enhanced chemiluminescent (ECL) detection system, following the manufacturer's instructions (ECL; GE Healthcare Life Sciences, Little Chalfont, UK). Image J software (NIH) was used for grey value analysis.

The article "Expression and clinical significance of hypoxia-inducible factor 1α, Snail and E-cadherin in human ovarian cancer cell lines" was retracted in 2025. Reasons: plagiarized data; overlap with other authors' work; concerns about the data.

### Immunohistochemistry

Streptvidin-peroxidase two-step immunohistochemical staining was performed in paraffin block of filed case; the experimental procedure was conducted in accordance with the manufacturer's instructions. Instead of the primary antibody, phosphate-buffered saline (Invitrogen Life Technologies) was used for the negative control while a known positive slide was used as the positive control.

### Evaluation of immunohistochemical staining

HIF-1α and Snail proteins are predominantly localized in the nucleus, occasionally accompanied by cytoplasmic staining. Endometrial glandular epithelial cells was predominantly localized to the nucleus and clear staining were selected as positive samples. Staining was graded as follows (13): i) Percentage of positively stained cells ≤5%, 0 points; 6–25%, 1 point; 26–50%, 2 points; 51–75%, 3 points; and 75%, 4 points. ii) Staining intensity was graded as: Colorless, 0 points; pale yellow, 1 point; brown, 2 points; and tan, 3 points. Samples in which the multiplication of the scores for the percentage of positively stained cells and the staining intensity resulted in values <2 were classified as negative expression and those ≥2 were classified as positive expression. E-cadherin protein was predominantly localized in the cell membrane, and E-cadherin expression in normal endometrial tissue was used as a positive control. In cancer cells, E-cadherin staining was graded as follows (11): No staining or positive staining rate ≤l0%, 0 points; low staining and positive staining rate ≥10, 1 point; moderate staining and positive staining rate ≥10, 2 points; staining as in normal tissue, classified as a high degree of staining, with a positive staining rate ≥10, 3 points. In order to simplify the statistical analysis, 0, 1 and 2 points were classified as reduced E-cadherin expression (reduced expression) and 3 points was classified as normal E-cadherin expression (preserved expression).

The article "Expression and clinical significance of hypoxia-inducible factor 1α, Snail and E-cadherin in human ovarian cancer cell lines" was retracted in 2025. Reasons: plagiarized data; overlap with other authors' work; concerns about the data.

### Statistical analysis

SPSS software, version 13.0 (SPSS, Inc., Chicago, IL, USA) was used for statistical analysis. The data are expressed as the mean ± standard deviation of 'n' experiments/samples. The comparison of numerical data was conducted using the χ^2^ test or Fisher's exact test and correlation analysis was performed using Spearman's rank correlation analysis. A two*-*tailed P<0.05 was considered to indicate a statistically significant difference.

## Results

### Invasiveness varies among ovarian cancer cell lines

The number of invasive cells in the human serous ovarian cancer cell line SKOV3 (132.6±6.4) and the human clear cell ovarian cancer cell line ES-2 (130.4±5.6) was significantly higher than that in the human undifferentiated ovarian cancer cell line TYK (102.3±4.7) and the human mucinous ovarian cancer cell line 3AO (104.1±5.2) (P<0.01).

### mRNA expression of HIF-1α and Snail is high and that of E-cadherin is low in invasive ovarian cancer cell lines

The mRNA expression levels of HIF-1α and Snail were greater in the highly invasive ovarian cancer cell lines SKOV3 and ES-2 as compared with those in the TYK and 3AO cell lines (104.1±5.2; P<0.01; Fig. 1). By contrast, the mRNA expression levels of E-cadherin were significantly lower in the SKOV3 and ES-2 cell lines than those in TYK and 3AO (P<0.05), as presented in Table II and Fig. 2.

### Protein expression of HIF-1α and Snail is high, while that of E-cadherin is low in invasive ovarian cancer cell lines

The protein expression levels of HIF-1α and Snail were greater in the highly invasive ovarian cancer cell lines SKOV3 and ES-2 than those in TYK and 3AO. By contrast, the expression levels of E-cadherin protein in SKOV3 and ES-2 were significantly lower than those in TYK and 3AO (P<0.05), as presented in Table III and Fig. 3. The results regarding protein expression were consistent with those of gene expression.

### HIF-1α, Snail and E-cadherin expression are correlated with clinicopathological factors of ovarian cancer

HIF-1α expression was significantly correlated with histological grading, tumor myometrial invasion, type of tissue and lymph node metastasis (P<0.05). Positive expression of Snail was closely correlated with surgical pathology stage, type of tissue and lymph node metastasis (P<0.05). Reduced expression of E-cadherin was significantly correlated with the histological type of tissue, tumor myometrial invasion and lymph node metastasis (P<0.01), as presented in Table IV and Figs. 4–6.

### Significant correlation between HIF-1α, Snail and E-cadherin expression in ovarian cancer tissues

The expression levels of HIF-1α and Snail in ovarian cancer exhibited a positive correlation (r=0.231; P=0.021), whereas the expression levels of Snail and E-cadherin were negatively correlated (r=−0.225; P=0.028), as presented in Table V, and there was a negative correlation between HIF-1α and E-Cadherin (r=−0.306; P<0.05).

The article "Expression and clinical significance of hypoxia-inducible factor 1α, Snail and E-cadherin in human ovarian cancer cell lines" was retracted in 2025. Reasons: plagiarized data; overlap with other authors' work; concerns about the data.

## Discussion

Cancer metastasis requires the occurrence of a primary tumor, local invasion and the formation of metastasis, involving a variety of molecular mechanisms which have remained to be fully elucidated to date. Thus, the clarification of these molecular mechanisms is an important challenge in cancer research (14).

A previous study identified that HIF-1α serves a critical role in the process of tumor adaptation to hypoxia (15), and HIF-1α expression was shown to be closely associated with tumor proliferation, invasion, metastasis, patient prognosis and resistance to treatment (16). In a study on ovarian cancer, Imai *et al* (7) demonstrated that the HIF-lα content of SKOV3 and OVCAR3 cells was upregulated following culturing under hypoxic conditions (5% oxygen) for 72 h. In addition, the invasiveness and metastatic potential were increased, accompanied by a significant increase in Snail gene expression and a significant reduction in E-cadherin gene expression, while normal ovarian epithelial OSE cells exhibited no such alterations. Immunohistochemical analysis demonstrated that high protein expression of HIF-lα in ovarian cancer tissue was associated with the lack of expression of E-cadherin (17,18). However, studies have also demonstrated that mRNA expression of HIF-lα in ovarian cancer and breast cancer exhibited no significant correlation with tumor grade, clinical stage and the survival rate (17,18). Yang *et al* (19) identified that overexpression of HIF-1α inhibits E-cadherin expression to promote the occurrence of EMT, which is mediated by Twist. The present study demonstrated that the protein and gene expression levels of HIF-1α in ovarian cancer cells were as follows: SKOV3 > ES-2 > 3AO > TYK (P<0.01), with the positive expression being significantly increased in specimens with lymph node metastasis. The expression levels of the Snail gene in ovarian cancer cells were as follows: SKOV3 = ES-2 > 3AO > TYK and the expression levels of Snail protein in ovarian cancer cells were as follows: ES-2 > SKOV3 > 3AO > TYK. The expression of Snail was in parallel with increases in HIF-lα, exhibiting a significant positive correlation in ovarian cancer (r=0.231; P=0.021). In addition, the present study revealed that HIF-1α protein expression was significantly correlated with histological grading, tumor myometrial invasion, tissue type and lymph node metastasis (P<0.05), which indicated that HIF-1α is involved in malignant processes of ovarian cancer development and progression and is closely correlated with invasion and metastasis.

The article "Expression and clinical significance of hypoxia-inducible factor 1α, Snail and E-cadherin in human ovarian cancer cell lines" was retracted in 2025. Reasons: plagiarized data; overlap with other authors' work; concerns about the data.

Kurrey *et al* (20) demonstrated that ovarian cancer cells transfected with exogenous Snail were able to undergo EMT, following which the cell invasiveness and motility were observed to be increased. This suggested that the transcription factor Snail has an important role in the process of metastasis in ovarian cancer. Snail expression has been demonstrated to be significantly associated with clinicopathological tumor staging, with a previous study identifying that Snail was associated with lymph node metastasis (20). An additional study observed that high Snail expression was closely associated with tumor recurrence and poor prognosis (21,22). Blechschmidt *et al* (13) demonstrated, through immunohistochemical analysis of Snail and E-cadherin in 48 cases of primary ovarian cancer and metastatic cancer, that the expression of Snail was significantly associated with E-cadherin expression in the primary tumor and metastasis of ovarian cancer. E-cadherin expression was significantly reduced in primary cancer tissues, while Snail expression was significantly increased. Their expression levels were observed to be significantly correlated with clinicopathological staging and a poor prognosis of ovarian cancer, and the expression trend was more marked in the metastatic cancer. In a study on 95 patients with epithelial ovarian cancers, Yoshida *et al* (23) observed that, as benign ovarian epithelial cells progressed into borderline tumors and then to ovarian cancer, Snail protein expression was gradually increased, whereas the expression levels of E-cadherin continued to decrease. In analogy with these results, the present study identified an inverse correlation between the expression of Snail and E-cadherin (r=−0.225; P=0.028), positive expression of Snail was significantly correlated with surgical stage, histological type and lymph node metastasis (P<0.05), while negative expression of E-cadherin was significantly associated with histological type, tumor myometrial invasion and lymph node metastasis (P<0.01). Based on previous studies and the results of the present study, E-cadherin is likely to be a direct target of Snail, serving an important role in invasion and metastasis in ovarian cancer.

HIF-1α may inhibit the expression levels of E-cadherin by upregulating the expression of Snail, serving an important role in invasion and metastasis in ovarian cancer. The results of the present study lead to the hypothesis that as a transcription factor, Snail is at the center of a signaling pathway cascade (HIF-1α regulates Snail, which in turn regulates E-cadherin), regulating upstream signal transduction pathways and downstream Snail transcriptional regulation of gene expression. It was suggested that the degree of malignancy of ovarian cancer can be reduced by blocking the Snail signaling pathway, reducing the invasive and metastatic potential of the tumor cells, thereby improving the prognosis of the patients. In addition, Snail is a potential tumor marker for metastatic potential, which may aid in the development of novel tumor treatment strategies and improve survival rates of patients with ovarian cancer.

The article "Expression and clinical significance of hypoxia-inducible factor 1α, Snail and E-cadherin in human ovarian cancer cell lines" was retracted in 2025. Reasons: plagiarized data; overlap with other authors' work; concerns about the data.

## Figures and Tables

**Figure 1:** Results of invasion assay indicating that SKOV3 cells (132.6±6.4) and ES-2 cells (130.4±5.6) had a much higher metastatic potential than TYK cells (102.3±4.7) and 3AO cells (104.1±5.2).

**Figure 2:** mRNA expression of the HIF-1α, Snail and E-cadherin genes in ovarian cancer cells. Reverse transcription polymerase chain reaction analysis of HIF-1α, Snail and E-cadherin in TYK, ES-2, SKOV3 and 3AO ovarian cancer cell lines; GAPDH levels were used as control for integrity of RNA samples. HIF-1α, hypoxia-inducible factor-1α.

**Figure 3:** Protein expression of HIF-1α, Snail and E-cadherin in ovarian cancer cells. Western blot analysis of HIF-1α, Snail and E-cadherin in SKOV3, ES-2, 3AO and TYK ovarian cancer cells. Equal loading of protein was confirmed by GAPDH. HIF-1α, hypoxia-inducible factor-1α.

**Figure 4:** Immunohistological analysis of HIF-1α protein in ovarian cancer tissue (magnification, x100). HIF-1α, hypoxia-inducible factor-1α.

**Figure 5:** Immunohistological analysis of Snail protein in ovarian cancer tissue (magnification, ×100).

**Figure 6:** Immunohistological analysis of E-cadherin protein in ovarian cancer tissue (magnification, ×100).

**Table I:** Polymerase chain reaction primers.

Protein	Primer sequences	Gene length (bp)
Snail	F: 5′-ATGCATGACCGGACACACCCATTAC-3′	2048
	R: 5′-AGATTTATTCTGCATCTGAATGCTC-3′	
E-cadherin	F: 5′-AAGTGCTGCCACCAAAGACAGA-3′	1581
	R: 5′-AGGTCAAGGCACCTCAATCATCCTC-3′	
HIF-1α	F: 5′-TGATACCAAAACCAATACACCTC-3′	2472
	R: 5′-TGCTGAATTCACACAGTCACAAC-3′	
GAPDH	F: 5′-ATTCCATGGCACCGTCAAGGCT-3′	527
	R: 5′-TCAGGTCCACCACTGACACGTT-3′	

HIF-1α, hypoxia-inducible factor 1α; bp, base pairs.

**Table II:** mRNA expression levels of the HIF-1α, Snail and E-cadherin genes in ovarian cancer cells.

Ovarian cancer cell line	HIF-1α/GAPDH	Snail/GAPDH	E-cadherin/GAPDH
3AO	0.64±0.12	0.56±0.08	1.11±0.15
SKOV3	1.22±0.25	1.17±0.20	0.48±0.08
ES-2	0.98±0.18	1.14±0.18	0.45±0.06
TYK	0.47±0.08	0.92±0.17	1.37±0.26

HIF-1α, hypoxia-inducible factor 1α.

**Table III:** Protein expression levels of HIF-1α, Snail and E-cadherin in ovarian cancer cells.

Types of ovarian cancer	HIF-1α/GAPDH	Snail/GAPDH	E-cadherin/GAPDH
3AO	0.87±0.13	0.65±0.10	1.12±0.21
SKOV3	1.25±0.22	1.34±0.27	0.71±0.17
ES-2	1.79±0.45	1.87±0.51	0.88±0.11
TYK	0.36±0.05	0.45±0.09	1.16±0.23

HIF-1α, hypoxia-inducible factor 1α.

The article "Expression and clinical significance of hypoxia-inducible factor 1α, Snail and E-cadherin in human ovarian cancer cell lines" was retracted in 2025. Reasons: plagiarized data; overlap with other authors' work; concerns about the data.

**Table IV:** Associations between expression of HIF-1α, Snail and E-cadherin in ovarian cancer and clinical pathological factors.

Clinical factors	Cases (n)	HIF-1α			Snail			E-cadherin		
		(−)	(+)	P	(−)	(+)	P	(−)	(+)	P
Age (years)				>0.05			>0.05			>0.05
<50	47	16	31		27	20		30	17	
≥50	135	57	78		71	64		89	46	
Histological grade				<0.05			>0.05			>0.05
I	80	42	38		48	32		53	27	
II	57	20	37		26	31		37	20	
III	45	11	34		24	21		29	16	
FIGO stage				>0.05			<0.05			>0.05
I+II	148	67	81		92	56		96	52	
III+IV	34	6	28		6	28		23	11	
Type of tissue				<0.05			<0.05			<0.01
Mucinous	53	29	24		43	10		30	23	
Serous	78	24	54		28	50		64	14	
Clear cell	21	6	15		7	14		15	6	
Undifferentiated	30	14	16	<0.05	20	10		10	20	
Myometrial invasion							>0.05			<0.01
<1/2	125	59	66		75	50		62	53	
≥1/2	57	14	43		23	34		47	10	
Lymph node metastasis				<0.05			<0.05			<0.01
No	136	63	73		87	49		81	55	
Yes	46	10	36		11	35		38	8	

FIGO, international federation of gynecology and obstetrics. HIF-1α, hypoxia-inducible factor 1α.

**Table V:** Correlation between Snail and HIF-1α/E-cadherin in ovarian cancer tissue.

Snail	Cases (n)	HIF-1α		Spearman		E-cadherin		Spearman	
		(−)	(+)	r	P	(−)	(+)	r	P
Negative	98	49	47			57	42		
Positive	84	24	62	0.231	0.021	62	21	−0.225	0.028

HIF-1α, hypoxia-inducible factor 1α.
